This article has been retracted.

# A wireless soil moisture sensor powered by solar energy

**DOI:** 10.1371/journal.pone.0184125

**Published:** 2017-09-08

**Authors:** Mingliang Jiang, Mouchao Lv, Zhong Deng, Guoliang Zhai

**Affiliations:** 1 Farmland Irrigation Research Institute, Chinese Academy of Agricultural Sciences, Muye District, Xinxiang City Henan province, China; 2 Key Laboratory of Water-Saving Agriculture of Henan Province, Muye District, Xinxiang City Henan province, China; 3 Center for Efficient Irrigation Engineering and Technology Research, CAAS, Muye District, Xinxiang City Henan province, China; Universita degli Studi della Tuscia, ITALY

## Abstract

In a variety of agricultural activities, such as irrigation scheduling and nutrient management, soil water content is regarded as an essential parameter. Either power supply or long-distance cable is hardly available within field scale. For the necessity of monitoring soil water dynamics at field scale, this study presents a wireless soil moisture sensor based on the impedance transform of the frequency domain. The sensor system is powered by solar energy, and the data can be instantly transmitted by wireless communication. The sensor electrodes are embedded into the bottom of a supporting rod so that the sensor can measure soil water contents at different depths. An optimal design with time executing sequence is considered to reduce the energy consumption. The experimental results showed that the sensor is a promising tool for monitoring moisture in large-scale farmland using solar power and wireless communication.

## 1. Introduction

Soil water content plays an important role in governing crop growth and yield. The serious water shortage in Northern China requires a more efficient way of agricultural water resources development. In recent years, the soil-based water measurements is used in a various devices[1–4]. These techniques provide farmers with information about the most appropriate volumes of irrigation to apply in each phenological period of the crop. There is a wide range of electrically based soil moisture measurement techniques established in the fields of geophysical surveying [5–6] and agronomy[7–9]. These include resistivity based methods[10–11]; capacitance based methods such as Frequency Domain Reflectometry (FDR)[12]; Time Domain Reflectometry (TDR)[13]; as well as Radiation based techniques[14]. Although low cost implementations of resistive based sensors have been suggested in the past[15–16], commercial implementations of these devices (for example the Landmapper^®^, that include interpretation software for vertical electrical properties of the soil) are expensive (typically $500–$1600), lack integrated data-logging capabilities, or are simply unavailable. Nowadays, with the rapid development of information and communication technology, Wireless Sensor Network (WSNs), as a new information acquisition and processing technology, has been widely used in real life[17–18].

To monitor soil water content dynamically in the farmland, a sensor technique, which has high accuracy and rapid response, low energy consumption and cost, is desired[19–20]. In early times, techniques for this purpose were a plaster sensor and tensiometer, but their response was unsatisfactory and there was hysteresis error between wetting and drying[21]. Since Topp [22]presented a three-order polynomial equation to approximate the relationship between the volumetric soil water content (VSWC) and relative dielectric constant of moist soil, many kinds of dielectric sensors based on TDR and FDR principles have been developed[23–26]. TDR sensors take a number of seconds to complete a water content measurement[27]. A more rapid response can be achieved by FD sensor, which only needs a fraction of a second[28]. However, there still have two technique limitations: 1) Underground power supply cables are impractical under large farmland areas, and the life of batteries is limited. The energy consumption, environmental and human labor costs required to change batteries regularly for a soil moisture sensor network to be used in an irrigation system are prohibitive. Providing a stable and lasting energy supplement for sensors by solar power must be considered. 2) Because the sensor output signals transmitted by long-distance cables are unrealistic in a farmland environment[29], so another limitation is to wirelessly transfer the data with data-loggers or routers across a certain distance.

In this study, we developed a soil moisture sensor that does not require external cables but rather uses a solar battery for power supply and a wireless transceiver module for data transmission, and then a field evaluation was conducted. The manuscript includes, firstly, the description of the electrical methods that are used to determine soil water content for sensor system. Moreover, the description experiments to illustrate the calibration equation of water content sensor in the designed sensor system. Subsequently, the obtained results in the cited experiments are discussed. Finally, some conclusions about the experiments and the possibilities of the employment of this device for irrigation management are added.

## 2. Materials and methods

### 2.1 General description of the designed system

Fig 1 schematically shows the designed system, which including a solar panel (multi-crystalline silicon, diameter 170mm), a supporting rod (stainless steel, diameter 10mm, length 600mm), a soil water content sensor and a wireless communication module (nRF905, Nordic, Norway). Besides, a micro-controller (MSP430F149) together with an extended memory chip (FLASH, 1MB) used as a data-logger. Different sources of energy exist in different forms (e.g. light, vibration, and electromagnetic waves). These sources can be harvested and used to extend battery life of a sensor node[30]. To avoid the data loss in wireless transmission owing to occasional accidents, the data was also saved as back up in the memory chip. A major feature of this configuration was to allow for simple setting at a range of depth (100–500mm) and replacement in the field. The two electrodes of the sensor were embedded in the end of the supporting rod to measure the soil moisture. To make the sensor easily accessible in the soil, one of the electrodes has a conical shape, and the other electrode is annular, with a PVC insulation isolation ring between the two electrodes. The supporting rod is a hollow structure and contains a coaxial cable connecting the two electrodes. The soil moisture sensor circuit, information acquisition unit and wireless transceiver module are protected inside a plastic shield to avoid water and dust under farmland. To provide electric power, 4 batteries (Ni-MH, AA 1.5V, 2000mAh), recharged by solar energy, were used in series. The soil moisture sensor system can cost less than 57 USDs including solar power system, supporting rod (stainless steel), Frequency Domain probes, LP2981 level converter, electronic interfaces and MSP430F149 microcontroller. Table 1 summarizes the cost details of the soil moisture sensor system in this study.

**Fig 1:** Layout of solar-powered wireless sensor.

**Table 1:** Cost details of system.

Items	Number	Price/USDs
**Solar power system**	1	15
**Sensor circuit**	1	10
**Supporting rod**	1	8
**FD probe**	2	4
**Wireless transceiver module**	1	20
**Total**	6	57

As shown in Table 2, represented by any single model from different companies, some existing soil moisture sensors are listed and compared with the new sensor system in this study from view of cost and wireless network application. Featuring low-cost, energy efficiency and ease-of-use, for the most common sensors shown in Table 2, the new sensor system in this study show advantages over the other sensors.

**Table 2:** Comparison with other existing sensors.

	Tektronix TDR	TDR100	Acclima TDT	CS 616	ECH2O	New sensor
**Principle of operation**	TDR	TDR	TDT	TLO	Capacitance	FDR
**Sensor cost/USDs**	11700	3710	350	150	100	57
**Equipment required**	analysis software	data logger, analysis software	custom controller, custom software	data logger	data logger, custom controller, custom software	data logger, custom controller,

Table 3 summarizes the power consumption of each component. Because the operating current of the micro-controller was considerably lower (0.01mA), it was reasonably disregarded when compared to the power consumption of other components. To ensure that the system has the smallest power consumption, the sensor could be switched from operating mode to stand-by mode at different intervals, as required. In the stand-by mode, the soil moisture sensor, information acquisition unit and wireless transmission module have a power consumption of approximately zero. Activation is achieved by timing activation and random activation, and the interval of timing activation can be changed through the parameter settings. For example, during rainfall time, soil moisture changes rapidly, and the interval of timing activation can be reduced appropriately. Solar power cannot guarantee real-time charging during rainfall and creates a discrepancy between energy supply and demand. The solution to this problem is to gradually extend the activation interval once the MCU detects soil moisture close to the saturation point to ensure the effective use of battery energy. Random activation can be initiated by the external artificial launch activation signal, and the nRF905 receives this signal and then activates the MCU and soil moisture sensors and sends the measurement data in time. Furthermore, before nightfall, when the MCU detects that solar energy is not sufficient to maintain the power consumption of the controller itself, the charge controller is turned off such that the power consumption of this part falls to zero. Because the wireless transceiver module and MCU have different operating level requirements, a level converter LP2981 must be used. The rationality of the photoelectric conversion element is one of the main features of this system. In this research, the main performance parameters of the polysilicon solar panels are an open circuit voltage of 11 V, a short-circuit current of 37 mA, a working voltage of 9 V, and an operating current of 22 mA. We selected the nickel-metal hydride battery pack with an output voltage of 6 V and a discharge capacity of 2,100 mAh.

**Table 3:** Power consumption of system.

	working voltage/V	working current/mA
**Micro-controller**	3.3	0.01
**Soil moisture sensor**	6.0	25
**FLASH**	3.3	15(write), 4(read)
**DC-regulator**	6.0	1
**Wireless transceiver module**	3.3	12.5 (emitting), 11 (receiving)
**Recharge control unit**	6.0	2 (self-consumption)

During this experiment, the measurement interval was every 15min. As presented in Fig 2, the executing sequence of the system in the operating mode took 12s for a sampling process. According to the current consumption of each component shown in Table 1 and the executing sequence in Fig 2, the average current consumption of the system was equal to 3.2mA, in which 3mA resulted from the self-consumptions of DC-regulator (1mA) and recharge control unit (2mA). Since only 0.2mA comes from the current consumption of sampling process, which means 93.75% of total current consumption was due to the DC-regulator and recharge control unit.

**Fig 2:** Layout executing sequence of a sampling process in the sensor system. To = overall operating time, Tw = time to measure soil water content, T_d_ = delay time in between, Ts = time to send data, T_F_ = time to write data into FLASH.

### 2.2 Soil moisture sensor

Fig 1 shows two electrodes (a metallic ring and tip) of a capacitor that was embedded at the bottom of the supporting rod. The soil particles surrounding the electrodes created a dielectric material of the fringe-capacitance sensor. A segment of coaxial line connected the electrodes to the high-frequency oscillator (100MHz) through the center of the rod. The principle of operation of the Frequency Domain capacitance probe relies on the fact that the dielectric constant between water and air differs by a factor of 80. Thus the presence of water in the soil between the probe plates produces a highly significant change in its capacitance, the higher the water concentration, the higher the capacitance. Therefore the capacitance or dielectric constant of soil could be measured, and converted into VSWC via a specific calibration. As the probe is electrically insulated, there is no direct current flow within the soil, and thus the conductive effect of ion based salts in the soil is minimized. However different soil types can be expected to display different properties[31]. We adopted the FD-based impedance measurement method in this research. Fig 3 shows a schematic of the principle of the soil moisture sensor.

**Fig 3:** Schematic diagram of the soil water content sensor.

In Fig 3, the field effect of a soil moisture sensor is shown as the edge effect of the electric field distribution. The high-frequency impedance *Z*_*p*_ of the electrode is a function of soil moisture near the field. Although the impedance detection circuit cannot be embedded in the support bar, according to Eq (1) for transmission line theory via coaxial line impedance mapping, a slight change in the impedance Z_p_ can still be transmitted to the detection circuit.

$$Z_{T}\left(L\right)=Z_{C}\frac{Z_{P}+jZ_{C}\text{tan}\frac{2\pi f}{C}\sqrt{E}L}{Z_{C}+jZ_{P}\text{tan}\frac{2\pi f}{C}\sqrt{E}L}$$ (1)

where *Z*_*T*_ is the transform impedance of the transmission line; *Z*_*C*_ is the characteristic impedance of the transmission line, which depends on the structure of the transmission line; *f* is the operating frequency of the sensor; ℰ is the relative permittivity of the insulating material in the coaxial line; *L* is the length of the coaxial line; and *C* = 3 × 10^8^ *m*/*s*, which is electromagnetic wave propagation velocity in vacuum. Therefore, assuming that

$$L\frac{2\pi f}{C}\sqrt{\varepsilon }=\pi$$ (2)

which is

$$L=\frac{C}{2f\sqrt{\varepsilon }}=\frac{\lambda }{2\sqrt{\varepsilon }}$$ (3)

then we can conclude that

$$\;Z_{T}\left(\frac{\lambda }{2\sqrt{\varepsilon }}\right)=Z_{P}$$ (4)

Eq (4) shows that fidelity mapping of the impedance can be achieved when the length of coaxial line *L* satisfies Eq (4). Furthermore, from Fig 2,

$$Z_{P}=\frac{U_{b}}{U_{a}-U_{b}}Z_{0}$$ (5)

where *Z*_0_ is the circuit matching impedance. Eq (5) indicates that *Z*_*P*_ is measurable, it is still necessary to calibrate the sensor with soil samples of different water contents to obtain the quantitative relationship between *Z*_*P*_ and the volumetric water content.

In this study, the geometrical structure and dimension of both electrodes approximated to the design of the combined penetrometer. Because this sensor had a rapid response (a fraction of 1s) immediately after electrical power switched on, the operating duration was chosen within 5s (Fig 4) for a reliable measurement.

**Fig 4:** Schematic diagram of data acquisition and wireless transmission.

### 2.3 Information collection and wireless data transmission

The moisture sensor information acquisition unit is indicated by the dashed box section in Fig 4. The core chip is a TI MSP430F149 microcontroller. The microcontroller was chosen not only because it contains hardware resources (including 2KRAM, 12-bitA/D) that are able to meet the monitoring requirements of the sensor but also because it works in different modes corresponding to the desired ultra-low power operation (0.1–400 μA). Fig 4 shows that the moisture electrode signals are converted into digital signals by A/D; then, the digital signals are sent to the wireless transmission module nRF905 through the SP11 interface. The system is equipped with a dedicated internal backup battery to avoid data loss caused by solar battery failure. When the microcontroller detects a shortage of solar energy, it can enable the backup battery.

We considered power consumption and transmission distance when selecting a wireless transmission module. The operating level of nRF905 is 1.9–3.3 V. The operating frequency of the transmit/receive module can be selected from 433, 868, or 915 MHz The wireless transmission module can complete the processing header and cyclic redundancy check code automatically, relying on on-chip hardware to achieve Manchester encoding/decoding. The maximum transfer rate is 100 kbps, and the maximum data transfer is 32 bytes at a time. Under an output power of -10 dBm, the current consumption is 11 mA when transmitting data, the current consumption is 12.5 mA when receiving data and the standby state is only 2 μA. According to the technical manual of the module, its effective distance for wireless transmission could reach 100 m for an output power of -10 dBm.

## 3. Results and conclusions

### 3.1 Calibration equation of water content sensor

Soil samples from the field were used for a site-specific calibration under laboratory conditions, prior to the field experiment, to ensure accurate measurements. To wirelessly collect data in the field, a central data-logger was set up for point to multi-point communication at a frequency bandwidth of 433.05–434.79MHz. After receiving the data from sensor, the central data-logger then transferred a data package to a PC via a standard USB port.

Fig 5 shows that the calibration results under the laboratory conditions fitted a quadratic equation (*R*^*2*^ = 0.9989) between the output of the fringe-capacitance sensor and VSWC ranging from dry to saturation (approximately 40%). This calibration outcome is closely agreed to that of the dielectric sensor that was integrated into a penetration rod[32].

**Fig 5:** Calibration results of the soil water content sensor.

### 3.2 Conclusions

The main purpose of the experiment was to test the feasibility of using this “plug-and-play” soil moisture sensor with a long-term solar power supply in the farmland environment. By interpreting the acquired data it is beneficial to better understand soil physical properties in the field and to manage the crop’s growing process for resource conservation. On the other hand, from the experiment overcomes related the solar panel size to the energy consumption, it is possible for the sensor to be miniaturized in physical dimension. The experiment results indicate that when sunlight is sufficient in Henan Province, the battery requires two days to fully charge in summer and 3 to 4 days to fully charge in winter. When the battery is fully charged, it can operate for 30 to 40 days continuously even after dynamic power is no longer added. Thus, we believe that this design is successful and can realize a "wireless" mode of soil moisture sensors for farm environments. Second, the experimental results show that the effective radius of the wireless data transmission is approximately 100 m, which lays a technical foundation for further research of wireless mesh water monitoring about large-area farmlands. Third, because this sensor can be inserted into different soil depths and provide real-time information about moisture distribution of different soil layers, it can be applied to various farmland irrigation automation systems. Thus, this sensor can be further developed as a node of wireless network at a field scale or be utilized individually in greenhouse.

## Supporting information

S1 File Basic datas of Fig 5. (XLSX)
